The article "CT-Assisted Improvements in the Accuracy of the Intraoperative Frozen Section Examination of Ground-Glass Density Nodules" was retracted in 2023. Reasons: unreliable results or conclusions; concerns about the data; concerns about the peer review; concerns about the citations.

# CT-Assisted Improvements in the Accuracy of the Intraoperative Frozen Section Examination of Ground-Glass Density Nodules

**DOI:** 10.1155/2022/8967643

**Published:** 2022-01-07

**Authors:** Wang Xinli, Sun Xiaoshuang, Yan Chengxin, Zhang Qiang

**Affiliations:** ^1^Department of Pathology, The Second Affiliated Hospital of Shandong First Medical University, Taian City, Shandong Province, China; ^2^Shandong First Medical University, Taian City, Shandong Province, China; ^3^Department of Medical Imaging, The Second Affiliated Hospital of Shandong First Medical University, Taian City, Shandong Province, China

## Abstract

**Objectives:**

The intraoperative frozen section examination (IFSE) of pulmonary ground-glass density nodules (GGNs) is a great challenge. In the present study, through comparing the correlation between the computed tomography (CT) findings and pathological diagnosis of GGNs, the CT features as independent risk factors affecting the examination were defined, and their value in the rapid intraoperative examination of GGNs was explored.

**Methods:**

The relevant clinical data of 90 patients with GGNs on CT were collected, and all CT findings of GGNs, including the maximum transverse diameter, average CT value, spiculation, solid component, vascular sign, air sign, bronchus sign, lobulation, and pleural indentation, were recorded. All the cases received thoracoscopic surgery, and final pathological results were obtained. The cases were divided into three groups on the basis of pathological diagnosis: benign/atypical adenomatous hyperplasia (AAH), adenocarcinoma in situ (AIS)/microinvasive adenocarcinoma (MIA), and invasive adenocarcinoma (IAC). The CT findings were analyzed statistically, the independent risk factors were identified through the intergroup bivariate logistic regression analysis on variables with statistically significant differences, and a receiver operating curve (ROC) was plotted to establish a logistic regression model for diagnosing GGNs. A retrospective analysis was conducted on the coincidence rate of the rapid intraoperative and routine postoperative pathological examinations of the 90 cases with GGNs. The relevant clinical data of 49 cases with GGNs were collected. Conventional rapid intraoperative examination and CT-assisted rapid intraoperative examination were performed, and their coincidence rates with routine postoperative pathological examinations were compared.

**Results:**

No statistical differences in the onset age, gender, smoking history, and family history of malignant tumors were found among cases with GGNs in the identification of benign/AAH, AIS/MIA, and IAC (*P* = 0.158, *P* = 0.947, *P* = 0.746, *P* = 0.566). No statistically significant difference was found among the three groups in terms of CT findings, such as lobulation, bronchus sign, pleural indentation, spiculation, vascular sign, and solid component (*P* > 0.05). The air sign, the maximum transverse diameter of GGNs, and average CT value showed statistically significant differences among the groups (*P* < 0.001, *P* < 0.05, *P* < 0.001). Bivariate logistic regression analysis was performed on three risk factors, and the predicted probability value was obtained. A ROC curve was plotted by using the maximum transverse diameter as a predictor for analysis between the groups with benign/AAH and AIS/MIA, and the results demonstrated that the area under the curve (AUC) was 0.692. A ROC curve was plotted by using the predicted probability value, maximum transverse diameter, and average CT value as predictors for distinguishing between the groups with AIS/MIA and IAC, and the results showed that the AUC values of the predicted probability value, maximum transverse diameter, and CT value were 0.920, 0.816, and 0.772, respectively. A regression model [Logit (*P*) = 2.304 − 2.689X1 + 0.302X2 + 0.011X3] was established to identify GGNs as IAC, obtaining AUC values of up to 0.920 for the groups with AIS/MIA and IAC, the sensitivity of 0.821, and the specificity of 0.894. The coincidence rate of rapid intraoperative and routine postoperative pathological examinations taken for modeling was 79.3%, that of conventional IFSE and postoperative pathological examination in prospective studies was 83.7%, and that of CT-assisted rapid intraoperative and postoperative pathological examinations was 98.0%. The former two were statistically different from the last one (*P* = 0.003 and *P* = 0.031, respectively).

The article "CT-Assisted Improvements in the Accuracy of the Intraoperative Frozen Section Examination of Ground-Glass Density Nodules" was retracted in 2023. Reasons: unreliable results or conclusions; concerns about the data; concerns about the peer review; concerns about the citations.

**Conclusion:**

The air sign, maximum transverse diameter, and average CT value of the CT findings of GGNs had superior capabilities to enhance the pathologic classification of GGNs. The auxiliary function of the comprehensive multifactor analysis of GGNs was better than that of single-factor analysis. CT-assisted diagnosis can improve the accuracy of rapid intraoperative examination, thereby increasing the accuracy of the selection of operative approaches in clinical practice.

## 1. Introduction

A ground-glass density nodule (GGN) manifests on computed tomography (CT) as a small region of pulmonary nodule with enhanced turbidity [1] and pathologically as an active inflammatory process or benign or malignant tumors [2]. With the popularity of low-dose CT, the detection rate of ground-glass lung nodules (GGNs) has increased annually, and a growing number of cases with early lung cancer have been screened out. According to the literature, the low-dose CT screening of patients with high risk of lung cancer can reduce the mortality of lung cancer by 20% [3].

The article "CT-Assisted Improvements in the Accuracy of the Intraoperative Frozen Section Examination of Ground-Glass Density Nodules" was retracted in 2023. Reasons: unreliable results or conclusions; concerns about the data; concerns about the peer review; concerns about the citations.

Surgical treatment has been always the most effective for lung cancer at the early stage. As a result of the two concepts of adenocarcinoma in situ (AIS)/microinvasive adenocarcinoma (MIA), as well as the technological advances in thoracoscopic surgery, the sublobectomy, including wedge resection and pulmonary segmentectomy, has a significant benefit in the treatment of early lung cancer [4]. The choice of pulmonary wedge resection, segmental resection, or pulmonary lobectomy is often based on the results of intraoperative frozen section examination (IFSE). However, the IFSE of pulmonary diseases always has some limitations. Firstly, pathologists can only collect 1–2 specimens from the lesion area, and the sampling range is very limited. Secondly, given the limitation of short diagnosis time, the production of frozen sections is not perfect, and the quality of tissue slices is often undesirable, and most importantly, numerous diagnostic traps are encountered in slicing, thus further complicating diagnosis. For GGNs, the differential diagnosis among atypical adenomatous hyperplasia (AAH), AIS, and MIA is dauntingly difficult, to identify whether there is invasion and the degree of invasion in the context of inflammation and fibrosis, to distinguish collapsed alveoli form adenoid structures against the backdrop of alveolar collapse, and to accurately distinguish true and false papillary structures are the key points in the diagnosis of GGNs of the lung and also a difficult problem for clinic pathologists.

In this study, the clinical characteristics and CT findings of 90 cases with GGNs were systematically reviewed, the correlation between CT findings and pathological diagnosis was statistically analyzed, a regression model for discriminating the differential diagnosis of GGNs was established, and prospective studies of 49 cases with GGNs were verified. The results of the present study showed that CT findings can assist in improving the accuracy of IFSE and offer good guarantees for precise treatment.

## 2. Materials and Methods

### 2.1. Subjects

Retrospective studies: the clinical data of 90 cases with GGNs on CT were collected, and they all admitted to the Department of Thoracic Surgery of the Second Affiliated Hospital of Shandong First Medical University from November 2017 to November 2020. The inclusion criteria were as follows [5]. All the cases received CT examination before surgery with, diagnosis of GGNs, and showed no distant metastasis [6]. The cases underwent thoracoscopic surgery and exhibited routine pathological results after surgery [2]. The maximum diameter of GGNs was less than or equal to 2 cm [7]. None of the cases received preoperative radiotherapy, chemotherapy, or any other treatment [4]. The clinical data of the cases were complete which included age, gender, smoking history, and family history of malignant tumors.

The article "CT-Assisted Improvements in the Accuracy of the Intraoperative Frozen Section Examination of Ground-Glass Density Nodules" was retracted in 2023. Reasons: unreliable results or conclusions; concerns about the data; concerns about the peer review; concerns about the citations.

*Prospective studies:* these studies included 49 cases with GGNs that were admitted to and received therapy by the Department of Thoracic Surgery from December 2020 to April 2021. The inclusion criteria were the same as those above.

All the cases provided signed informed consent, and the present study was also approved by the medical ethics committee of the hospital.

### 2.2. Histopathological Diagnosis

All tissue specimens were obtained through thoracoscopic surgery. Pathological sections for IFSE were produced routinely, and the pathological diagnosis was given by two senior pathologists. Specimens for routine postoperative pathological examinations were fixed in 10% neutral buffered formalin. The diagnosis was performed by two experienced pathologists. If diagnosis was difficult, immunohistochemistry was recommended for assistance. The pathological diagnosis covered benign lesions, including inflammation, cryptogenic organizing pneumonia, and granulomatous lesions: AAH; AIS; MIA; and invasive adenocarcinoma (IAC) (without distinguishing the histological subtypes of adenocarcinoma). All the cases were divided into three groups on the basis of pathological diagnosis: benign/AAH, AIS/MIA, and IAC.

### 2.3. CT Examination of GGNs

All the cases were examined by CT in our hospital. Philips Brilliance iCT (Netherlands) and GE Lihtspeed VCT (US) were adopted. Each case was instructed to lie on their back on the CT couch and to inhale deeply with both hands above their head. The CT was allowed to scan from the apex pulmonis to the basis pulmonis. A lung window (width: 1500 HU; level: −600 HU) was used. All diagnosis reports were completed by two radiologists, and the radiologic characteristics of each case were recorded. The CT findings of GGNs contained the maximum transverse diameter, lobulation, vascular sign, air sign, pleural indentation, spiculation, solid component, and average CT value.

### 2.4. CT-Assisted IFSE

The CT findings of the cases were analyzed before surgery, and the characteristics of GGNs were assessed by using the logistic regression model established in the present study. When the pathologic manifestations revealed in the IFSE were consistent with the assessment, the intraoperative pathological diagnosis was given. When the pathologic manifestations of rapid intraoperative examination were inconsistent with the CT-assisted preoperative assessment, the diagnosis was confirmed by reviewing specimens, repeated sampling and splicing, and discussion with additional individuals.

The article "CT-Assisted Improvements in the Accuracy of the Intraoperative Frozen Section Examination of Ground-Glass Density Nodules" was retracted in 2023. Reasons: unreliable results or conclusions; concerns about the data; concerns about the peer review; concerns about the citations.

### 2.5. Statistical Methods

By using SPSS19.0 software, the chi-square test was performed to compare the count data among the three groups, the univariate analysis was conducted on measurement data, and the *t*-test was carried out for between-group comparison. The between-group multivariate logistic regression analysis was performed for factors showing differences in the between-group comparison of the count and measurement data, and the predicted probability value was retained. By using the obtained factors with differences as the predictors, a receiver operating curve (ROC) was plotted to obtain the critical value, sensitivity, and specificity among groups. The chi-square test or Wilcoxon signed rank test was used for the comparison of the coincidence rate between intraoperative pathological diagnosis and final pathological diagnosis. A *P* value of less than 0.05 is considered statistically significant.

## 3. Results

### 3.1. Relationships between Clinical Features and Pathological Diagnosis

The average age of 90 cases with GGNs was 59.03 years old (37-84). Among the cases, 34 were males and 56 were females. A total of 21 cases had histories of smoking, and 5 cases had family histories of malignant tumors. The relationships among the ages, genders, smoking histories, family histories of malignant tumors, and routine pathological diagnoses of the 90 cases were analyzed. However, no significant difference was found (Table 1).

### 3.2. Relationships between CT Findings and Pathological Diagnosis

The maximum transverse diameter of the 90 cases with GGNs was 12.40 mm on average, fitted the normal distribution, and showed statistically significant differences in the comparison of the groups with benign/AAH, AIS/MIA, and IAC (*P* < 0.001) (Table 2). Differences between the groups with benign/AAH and AIS/MIA (*P* = 0.03) and those among the groups with benign/AAH, AIS/MIA, and IAC (*P* < 0.001) were statistically significant. These results suggested that the maximum transverse diameter of the lesion contributed to distinguishing the characteristics of GGNs.

The average CT value of 90 cases with GGNs was −489.58HU. Differences among the three groups were statistically significant (*P* < 0.001) (Table 2). Differences between the groups with benign/AAH and AIS/MIA were not statistically significant (*P* = 0.88). Differences between the groups with benign/AAH and AIS/MIA and the group with IAC were statistically significant (*P* < 0.001). This result suggested that the average CT value was helpful for distinguishing invasive carcinoma from the noninvasive lesions of GGNs.

The article "CT-Assisted Improvements in the Accuracy of the Intraoperative Frozen Section Examination of Ground-Glass Density Nodules" was retracted in 2023. Reasons: unreliable results or conclusions; concerns about the data; concerns about the peer review; concerns about the citations.

The groups with benign/AAH, AIS/MIA, and IAC were compared in terms of the relationships among lobulation, bronchus sign, pleural indentation, spiculation, air sign, vascular sign, and solid component, and only air sign showed differences (*P* < 0.001) (Table 2). Differences were observed between the groups with benign/AAH and AIS/MIA and the group with IAC (*P* = 0.017 and *P* < 0.001). However, no difference was observed between the groups with benign/AAH and AIS/MIA (*P* = 1.00). This result suggested that air sign was conducive to distinguishing invasive carcinoma from the noninvasive lesions of GGNs.

### 3.3. Analysis of the ROC Curves of the Maximum Transverse Diameter and Average CT Value

Bivariate logistic regression analysis was performed on the groups with benign/AAH and AIS/MIA by using the maximum transverse diameter, air sign, and average CT value as independent variables. The results are given in Table 3.

Bivariate logistic regression analysis was performed on the groups with AIS/MIA and IAC by using the maximum diameter, air sign, and average CT value as independent variables. The results are listed in Table 4.

Bivariate logistic regression analysis showed that the maximum transverse diameter of GGNs was an independent risk factor for determining the grouping of benign/AAH and AIS/MIA, whereas the maximum transverse diameter and the average CT value were independent risk factors for distinguishing between the groups with AIS/MIA and IAC. The ROC curves of the groups with benign/AAH and AIS/MIA were plotted with the maximum transverse diameter as the test variable (Figure 1) with the following results: critical value of 10.5 mm, area under the curve (AUC) of 0.692, sensitivity of 0.511, specificity pf 0.800, and Youden index of 0.311. These results suggested that the maximum transverse diameter of 10.5 mm was of predictive significance for distinguishing benign/AAH from AIS/MIA, but had low diagnostic value.

The ROC curves of the groups with AIS/MIA and IAC were plotted with the maximum transverse diameter of GGNs and the average CT value as predictors (Figure 2, Table 5). The results revealed that when the ROC curve was plotted with the maximum transverse diameter as the test variable, the AUC was 0.816, the sensitivity was 0.786, the specificity was 0.613, and the Youden index was 0.531, indicating that the maximum transverse diameter of 13.5 mm was of good predictive significance for distinguishing between the groups with AIS/MIA and IAC. When the ROC curve was plotted with the average CT value as the test variable, the AUC was 0.772, the sensitivity was 0.714, the specificity was 0.809, and the Youden index was 0.523, indicating that the average CT value of −446 HU had good predictive significance for distinguishing between the groups with AIS/MIA and IAC. The measurement data and the count data were comprehensively analyzed by using the bivariate logistic regression model, and a model [Logit (*P*) = 2.304 − 2.689X1 + 0.302X2 + 0.011X3] for distinguishing between the groups with AIS/MIA and IAC was obtained with the AUC of 0.920, the sensitivity of 0.821, the specificity of 0.894, and the Youden index of 0.715.1.

The article "CT-Assisted Improvements in the Accuracy of the Intraoperative Frozen Section Examination of Ground-Glass Density Nodules" was retracted in 2023. Reasons: unreliable results or conclusions; concerns about the data; concerns about the peer review; concerns about the citations.

### 3.4. Improvements in Diagnostic Coincidence Rate by CT-Assisted IFSE

A total of 87 out of the 90 cases with GGNs in the retrospective studies received IFSE. Among these cases, 69 had consistent diagnosis with routine pathological results, and 18 lacked diagnostic coincidence with the results; that is, the coincidence rate was 79.3%. Among the 46 cases in the group with AIS/MIA, 14 had inconsistent results from final pathological results, accounting for 30.4% of the group, and 8 out of the 14 cases were diagnosed with IAC (Figure 3). The data of a total of 49 cases with GGNs were collected in the prospective studies. The intraoperative pathological diagnosis for 8 cases that received conventional IFSEs did not match the findings of routine postoperative pathological examinations, and only 1 of the cases that underwent CT-assisted IFSE had the findings inconsistent with final diagnosis. As revealed in the retrospective and prospective studies, statistically significant differences existed between the groups diagnosed with conventional IFSE and CT-assisted IFSE in terms of diagnostic coincidence rate (*P* = 0.003 and *P* = 0.031), indicating that CT-assisted IFSE could improve the accuracy of intraoperative diagnosis and facilitate accurate treatment decision-making.

## 4. Discussion

Surgical treatment is the clinically preferred treatment for GGNs with imaging findings that tend to be malignant lesions. Sublobectomy as a surgical approach for the treatment of early lung cancer has risen significantly with advances in thoracoscopic surgery and the patients' appeal for good prognosis. However, considering problems, such as metastasis and recurrence, strict standards for sublobectomy exist, including AIS or IAC as the pathological result of IFSE. IFSE is pathologically limited by time and the number of specimens, and the diagnostic accuracy rate of this examination is often lower than that of routine postoperative pathological examinations. In 2012, Walts and Marchevsky [8] found that the coincidence rate of IFSE with routine postoperative pathological examinations is 68% when the diameter of the lung tumor is less than or equal to 1 cm, and the accuracy rate of IFSE is only 84.3% when the tumor diameter exceeds 1 cm. These low accuracy rates can be attributed to the underestimation of AIS and MIA in the IFSE. This situation is a common problem and a common challenge encountered by pathologists in quickly making the accurate pathological diagnosis of GGNs during the procedure.

The article "CT-Assisted Improvements in the Accuracy of the Intraoperative Frozen Section Examination of Ground-Glass Density Nodules" was retracted in 2023. Reasons: unreliable results or conclusions; concerns about the data; concerns about the peer review; concerns about the citations.

With the increasing popularity of low-dose CT, the number of cases that are being diagnosed in the early stage of lung cancer is growing [9]. Although CT findings are useful for assessing the malignant characteristics of GGNs to certain extent, criteria for specificity are lacking. The importance of CT findings, such as lobulation, bronchus sign, pleural indentation, spiculation, air sign, vascular sign, and solid component, in the identification of GGNs remains unclear; although, numerous studies have been done by many scholars [10]. The present study found that the air sign on CT was helpful for the differential diagnosis of benign/AAH, AIS/MIA, and IAC. Bivariate logistic regression analysis revealed that the air sign was an independent risk factor for predicting GGNs as IAC. The air sign usually occurs at the early stage of lung cancer. It is often manifested with alveolar ectasia and bronchiole distortion with peripheral tissues that are not destroyed by tumors. Consistent with our findings, the results of Zhan et al. [11] showed that the air sign is suggestive of the diagnosis of IAC. Although IAC frequently occurs with lobulation, pleural indentation, and spiculation, these characteristics are not significantly different when GGNs manifest with preinvasive lesions or MIA [7].

The present study found that the maximum transverse diameter and average CT value are valuable for the identification of GGNs. Nodule size is a useful parameter for evaluating the possibility of malignant tumors, and the possibility of malignant tumors gradually increases with the diameter of nodules. Fan et al. believed that the possibility of malignancy increases by 1.123 times for every 1 mm increase in nodule diameter [5]. Zhan et al. revealed that IAC is highly likely when the maximum diameter on thin-layer CT is 8.12 mm [11]. Zhang suggested that the diameter of GGNs in IAC is usually greater than or equal to 12.2 mm [12]. In the present study, differences were found among the maximum transverse diameters of the groups with benign/AAH, AIS/MIA, and IAC, and through the bivariate logistic regression analysis, the maximum transverse diameter was identified as an independent risk factor for distinguishing among the three groups. The optimal critical value of the maximum diameter of the groups with benign/AAH and AIS/MIA was 10.5 mm, and the AUC was 0.692 and insufficient to distinguish between the two groups. However, that of the groups with benign/AAH and IAC was 13.5 mm with the sensitivity of 0.786 and the specificity of 0.613, indicating a superior diagnostic value. These findings were consistent with the results of previous literature and reports, suggesting that the maximum diameter gradually increases with the malignancy of GGNs and can be used as a leading reference for the grouping of AIS/MIA and IAC. In the present study, differences among the average CT value of the three groups were statistically significant. As revealed through the bivariate logistic regression analysis, the average CT value was an independent risk factor for distinguishing between the groups with AIS/MIA and IAC. The optimal critical value of the groups with AIS/MIA and IAC was −446HU with the sensitivity of 0.714 and the specificity of 0.809. Therefore, the average CT value could be used as a reference index for distinguishing non-IAC from IAC. Likewise, Zhou et al. found that the average CT value of −583.60 HU (with the sensitivity of 68.8% and the specificity of 66.9%) is a differential index for distinguishing non-IAC from IAC [13]. Kitazawa reflected that −489 HU is an important predictor for IAC [6]. The increment in the CT value is usually believed to be the result of tumor cytosis [14].

The article "CT-Assisted Improvements in the Accuracy of the Intraoperative Frozen Section Examination of Ground-Glass Density Nodules" was retracted in 2023. Reasons: unreliable results or conclusions; concerns about the data; concerns about the peer review; concerns about the citations.

Among the 87 cases with GGNs in the retrospective studies, 18 had IFSE results that were inconsistent with postoperative pathological diagnosis. Among these cases, 8 with AIS and MIA were diagnosed as having IAC during the operation, which caused overdiagnosis. Evidently, during the diagnosis of GGNs, distinguishing AIS from MIA was the difficulty encountered in the rapid intraoperative examination of GGNs. In prospective studies, CT was used to assist in the analysis of GGNs before surgery. When the results of rapid intraoperative examination are inconsistent with the preoperative anticipation and the pathological results are difficult to diagnose, an appropriate method must be actively taken to reexamine, resample, and reslice specimens and discuss with additional individuals to avoid the misdiagnosis of some GGNs.

In summary, the present study found differences among the groups with benign/AAH, AIS/MIA, and IAC in terms of the CT manifestations of GGNs, such as air sign, maximum transverse diameter, and average CT value. The logistic regression model established in the present study can assist in the analysis of the pathological types of GGNs on CT and has greater value in assisting in the diagnosis than the independent use of a single factor. CT-assisted diagnosis can significantly improve the diagnostic accuracy of GGNs in IFSE, thereby improving the accuracy of surgical technique selection in clinical practice.

The article "CT-Assisted Improvements in the Accuracy of the Intraoperative Frozen Section Examination of Ground-Glass Density Nodules" was retracted in 2023. Reasons: unreliable results or conclusions; concerns about the data; concerns about the peer review; concerns about the citations.

## Figures and Tables

**Figure 1:** ROC curves of the groups with benign/AAH and AIS/MIA.

**Figure 2:** ROC curves of the groups with AIS/MIA and IAC.

**Figure 3:** Case diagnosed with IAC by IFSE (a) and with AIS by routine postoperative pathological examinations (b).

**Table 1:** Relationships between the clinical features and pathological diagnosis of 90 cases with GGNs.

Clinical features	Benign/AAH	AIS/MIA	IAC	Total	*P* value
Average age (years)	59.80 ± 9.59	57.26 ± 10.21	61.61 ± 8.22		0.158
Gender					0.974
Male	5	18	11	34	
Female	10	29	17	56	
Smoking history					0.746
Yes	4	9	8	21	
No	11	38	20	69	
Histories of malignant tumors					0.566
Yes	0	4	1	5	
No	15	43	27	85	

**Table 2:** Relationships between the CT findings and pathological diagnosis of the 90 cases with GGNs.

Clinical features	Benign/AAH	AIS/MIA	IAC	Total	*P* value
Maximum diameter of GGNs (mm)	8.60 ± 3.92	11.27 ± 4.28	16.16 ± 3.78		<0.001
Average CT value (HU)	−542.07 ± 91.83	−536.36 ± 140.25	−382.93 ± 148.23		<0.001
Lobulation					0.188
Yes	1	7	8	16	
No	14	40	20	74	
Bronchus sign					0.070
Yes	0	1	4	5	
No	15	46	24	85	
Pleural indentation					0.278
Yes	4	9	10	23	
No	11	38	18	67	
Spiculation					0.253
Yes	1	3	5	9	
No	14	44	23	81	
Air sign					<0.001
Yes	1	2	12	15	
No	14	45	16	75	
Vascular sign					0.052
Yes	3	12	14	29	
No	12	35	14	61	
Solid component					0.938
Yes	3	11	5	19	
No	12	36	23	71	

**Table 3:** Logistic regression analysis on the CT findings of the groups with benign/AAH and AIS/MIA.

Variables	*B*	SE	Wald	OR	*P* value	95% CI
Air sign	0.695	1.278	0.266	1.933	0.606	0.042–6.329
Maximum transverse diameter	0.186	0.091	4.163	1.204	0.041	0.695–0.993
Average CT value	0.001	0.002	0.090	1.001	0.764	0.995–1.004

**Table 4:** Logistic regression analysis on the CT findings of the groups with AIS/MIA and IAC.

Variables	*B*	SE	Wald	OR	*P* value	95% CI
Air sign (X1)	−2.689	1.032	6.794	0.068	0.009	0.009–0.513
Maximum transverse diameter (X2)	0.302	0.094	10.368	1.352	0.001	1.125–1.625
Average CT value (X3)	0.011	0.003	10.971	1.011	0.001	1.004–1.017

**Table 5:** ROC curves analysis of the groups with AIS/MIA and IAC.

	Critical value	Sensitivity	Specificity	AUC	Youden index
Maximum diameter (mm)	13.5	0.786	0.613	0.816	0.531
CT value (HU)	−446	0.714	0.809	0.772	0.523
Predicted probability value	0.1523	0.821	0.894	0.920	0.715

## Data Availability

The data used to support the findings of this study are available from the corresponding author upon request.
